# Efficacy and safety of traditional chemotherapies for patients with ovarian neoplasm: a network meta-analysis

**DOI:** 10.18632/oncotarget.16729

**Published:** 2017-03-30

**Authors:** Lili Yang, Gongliang Guo, Liqun Sun, Chenhao Li, Haipeng Zhang

**Affiliations:** ^1^ Department of Gynecology and Obstetrics, The First Hospital of Jilin University, Changchun, Jilin, China; ^2^ Department of Cardiology, China Japan Union Hospital Jilin University, Changchun, Jilin, China; ^3^ Outpatient Department of Pediatrics, The First Hospital of Jilin University, Changchun, Jilin, China; ^4^ Department of Nephropathy, The First Hospital of Jilin University, Changchun, Jilin China; ^5^ Department of Gynecology, The First Hospital of Jilin University, Changchun, Jilin, China

**Keywords:** ovarian neoplasm, network meta-analysis, carboplatin, pegylated liposomal doxorubicin, paclitaxel

## Abstract

**Background:**

Ovarian neoplasm is a kind of high risky cancer among female. This paper assessed the efficacy and safety of twelve therapies and figured out the superior chemotherapeutic drug for ovarian cancer through network meta-analysis (NMA).

**Method:**

Eligible randomized controlled trials (RCTs) were retrieved from electronic databases. Primary outcomes concerning efficacy, overall survival (OS) and progression-free survival (PFS), were presented as hazard ratio (HR) and the associated 95% credible interval(*CrI*), while outcomes concerning safety were assessed by odds ratio (OR) and the corresponding 95% *CrI*. Surface under the cumulative ranking curve (SUCRA) was calculated under each survival and safety outcome in order to show the rankings of tested therapies.

**Result:**

Electronic databases such as PubMed and Embase were searched to finally obtain 19 eligible studies of 16290 patients. In accordance of primary outcomes, when it came to 3-y PFS, paclitaxel/epirubicin/carboplatin (Pa/E/Ca) and pegylated liposomal doxorubicin/ paclitaxel/ carboplatin (PLD/Pa/Ca) were preferred compared to carboplatin (Ca) (HR= 0.80, 95% *CrI*= 0.67-0.96; HR= 0.83, 95% *CrI*= 0.69-0.99). According to 5y-PFS, Pa/E/Ca was notably better than Ca (HR= 0.80, 95% *CrI*= 0.65-0.99). As to adverse effects, Ca was superior to Pa/E/Ca in neuropathy (HR=0.05, 95% *CrI*=0.02-0.19). Pa/E/Ca showed high rankings in 3y-PFS (SUCRA=0.749), 5y-OS (SUCRA=0.738) and 5y-PFS (SUCRA=0.798) while (PLD/Pa/Ca) in 3y-OS (SUCRA=0.737), 5y-OS (SUCRA=0.687) and 5y-PFS (SUCRA=0.712). Besides, Pa/E/Ca ranked the third with a SUCRA of 0.661 in neutropenia.

**Conclusion:**

PLD/Pa/Ca, PLD/Ca and Pa/E/Ca are highly recommended as potential therapeutically choices for patients with ovarian cancer. But considering the lack of safety data for PLD/Pa/Ca, this intervention should be taken with caution.

## INTRODUCTION

Ovarian neoplasm is a kind of cancer that forms in an ovary. Although etiology of ovarian neoplasm is not completely understood, potential factors, including age, late childbearing, hormone therapy after menopause, fertility medication, and obesity may raise the incidence [1]. Most of the patients with ovarian neoplasm fail to be diagnosed at early stages [2]. According to a recent authoritative report, ovarian neoplasm accounts for 0.7% cumulative risk of incidence and 0.6% cumulative risk of death in more developed areas [3]. Also it has 0.5% cumulative risk of incidence and 0.4% cumulative risk of death in developing areas. Records suggest that every year 238,100 new cases and 151,900 deaths are estimated all over the world, making ovarian neoplasm the 8^th^ most dangerous cancer among women [4]. Thus it's necessary for researchers to screen out proper therapies treatments for patients with ovarian neoplasm.

The management of ovarian neoplasm usually involves chemotherapy and surgery. When it comes to more aggressive tumors, chemotherapy, especially combinations of chemotherapy regimens are preferred. For instance, both carboplatin and cisplatin are platinum-based therapies, while in the past carboplatin (Ca) is the most widely used therapy because of its less toxicity and relatively high activity [5]. Ca is accepted as a basic first-line treatment for ovarian neoplasm, and other different therapies are used in combination of Ca treatment for sake of achieving better efficacy. For example, paclitaxel was first tested in ovarian cancer in the early 1990s, while it plus carboplatin (Pa/Ca) performed good outcomes in terms of overall survival [6]; and irinotecan/ cisplatin (Ir/Ci) [7] is suggested to be an effective therapy against ovarian neoplasm. Moreover, other regimens contain Ca are also proved to be effective second-line therapies, such as interferon-alpha plus carboplatin (Ia/Ca) [8], epirubicin (E) with carboplatin and paclitaxel (Pa/E/Ca) [9] and docetaxel (D), a kind of taxane derived from a typical compound found in the taxus baccata. D/Ca [10] shows efficacy not only in ovarian cancer but also in other cancers like breast cancer. Topotecan, gemcitabine, and pegylated liposomal doxorubicin (PLD) are cytotoxic agents approved by US Food & Drug Administration (FDA) as monotherapies for ovarian neoplasm, and their combination with carboplatin (T/Ca, G/Ca, PLD/Ca) are shown to be safe and equally efficacious treatments for ovarian cancer [11–13].

A number of trials discuss the efficacy and safety of the above mentioned treatments, but inconsistent results had rendered the real efficacy of one typical drug ambiguous. For example, one study claimed that PLD/Ca produced equal efficacy to Pa/Ca [13], while another study concluded that PLD/Ca was not superior to Pa/Ca [14] and a third study suggested PLD/Ca was effective and warranted a phase three evaluation [15]. Also, direct evidence for treatment comparison is still insufficient. Besides, though there existed one network meta-analysis (NMA) study [16], it only focused on eight different chemotherapy regimens and didn't analyze hazard ratio concerning time period, it also neglected the adverse effects of chemotherapies. Thus, the aim of our study is to complete a NMA using current outcomes from analysis of MA and RCTs, therefore every two therapies with or without direct comparison can be rationally evaluated. Moreover, both efficacy and safety factors will be taken into account in order to form a comprehensive ranking of therapies for patients’ benefits.

## RESULTS

### Literature search and network

A total of 3086 records were obtained from database searching and 339 articles were available for full text and data assessment after primary screening. By excluding duplicates and irrelevant topics, the number of eligible articles dropped to 42. Then, each article was screened by reviewers to rule out studies with irrelevant outcomes. Finally 19 trials with 16,290 patients were accepted including one article containing two comparisons (Figure 1) [7–15, 17–26]. The characteristics of studies included in the NMA were shown in Table 1. Most of the trials set Pa/Ca as control group because it was the most widely used medicine therapy for ovarian neoplasm. Other therapies included PLD/Ca, G/Ca, G/Pa/Ca, T/Pa/Ca, D/Ca, Pa/E/Ca, Ca, Cy/D/Ci, Ia/Ca, and PLD/Pa/Ca. The network plot was performed in Figure 2. The size of the nodes indicated the sample size and each two nodes that had a direct comparison were shown by a line connection.

**Figure 1:** Flow diagram of included and excluded studies

**Table 1:** Study characteristics

Author, Year	Country	Follow-up/month	Sample Size	Comparision	Primary Outcomes							Adverse Effects					
					1y-OS	3y-OS	5y-OS	1y-PFS	3y-PFS	5y-PFS		Alopecia	Neutropenia	Nausea	Vomiting	Diarrhea	Neuropathy
Sugiyama 2016	Japan	44.3	619	Ir/Ci vs. Pa/Ca	√	√	√	√	√	√		√	√	√	√	√	√
Mahner 2015	Multiple	49	259	PLD/Ca vs. Pa/Ca	√	√	√	√	√			√	√	√	√	√	√
Pignata 2011	Italy	40	820	PLD/Ca vs. Pa/Ca	√	√	√	√	√	√		√	√	√	√	√	√
Gordan 2011	US	22	831	G/Ca vs. Pa/Ca	√	√	√	√	√	√		√	√	√	√		√
du Bois 2010	Multiple	49	1742	G/Pa/Ca vs. Pa/Ca	√	√	√	√	√	√		√	√	√	√	√	√
Pujade-Lauraine 2010	Multiple	22	973	PLD/Ca vs. Pa/Ca				√	√			√	√	√	√	√	√
Bolis 2010	Italy	NA	326	T/Pa/Ca vs. Pa/Ca	√	√	√	√	√	√			√	√	√		√
Bafaloukos 2010	Multiple	43.6	174	PLD/Ca vs. Pa/Ca	√	√	√	√	√	√		√	√		√	√	√
Alberts 2008	Multiple	22.5	61	PLD/Ca vs. Ca	√	√		√	√				√	√	√		
Mori 2007	Japan	30	29	D/Ca vs. Pa/Ca	√	√		√	√				√				√
Pfisterer 2006	Multiple	42	1308	T/Pa/Ca vs. Pa/Ca	√	√	√	√	√	√		√		√	√	√	√
du Bois 2006	Italy	NA	1282	Pa/E/Ca vs. Pa/Ca	√	√	√	√	√	√				√	√	√	√
Gonzalez-Martin 2005	Multiple	17	78	Ca vs. Pa/Ca	√	√	√	√	√			√		√	√	√	√
Vasey 2004	US	NA	1077	D/Ca vs. Pa/Ca	√	√		√	√					√	√	√	√
De Placido 2004	Italy	28	273	T/Pa/Ca vs. Pa/Ca	√	√	√	√	√	√							
Parmar 2003	Multiple	42	802	Ca vs. Pa/Ca	√	√	√	√	√	√		√			√		
ICON group 2002	Multiple	51	1421	Ca vs. Pa/Ca	√	√	√	√	√	√		√			√		√
		51	653	Cy/D/Ci vs. Pa/Ca	√	√	√	√	√	√		√			√		√
Bruzzone 1997	Multiple	13	111	Ia/Ca vs. Ca	√	√	√	√	√	√		√				√	√
Bookman 2009	Multiple	NA	3451	G/Pa/Ca vs. Pa/Ca vs. PLD/Pa/Ca vs. T/Pa/Ca	√	√	√	√	√	√							

Abbreviations: NA: Not available; OS: Overall survival; PFS: Progression-free survival; Ir: Irinotecan; Ci: Cisplatin; Pa: Paclitaxel; Ca: Carboplatin; PLD: Pegylated liposomal doxorubicin; G: Gemcitabine; T: Topotecan; D: Doxorubicin; Cy: Cyclophosphamide; Ia: Interferon-alpha; E: Epirubicin.

**Figure 2:** Network diagram of all included studies Each node represents a treatment type; the diameters of circles represents the number of people involved and the widths of lines between two nodes represents the number of study involved in the head-to-head comparison. Abbreviation: Ir: Irinotecan; Ci: Cisplatin; Pa: Paclitaxel; Ca: Carboplatin; PLD: Pegylated liposomal doxorubicin; G: Gemcitabine; T: Topotecan; D: Doxorubicin; Cy: Cyclophosphamide; Ia: Interferon-alpha; E: Epirubicin.

### Network comparison among therapies

Both 1y-OS and 3y-OS could be found in 19 comparisons out of 20, while 16 trials contained 5y-OS. According to Table 2 and Figure 3, no evidence showed there existed significant statistical significance among different therapies. The 5-y PFS data could be found in 14 trials, while all trials included 1-y PFS and 3-y PFS. The results of network comparisons were shown in Table 2 and Figure 3. As to 1y-PFS, Pa/Ca, PLD/Ca and T/Pa/Ca appeared to be more effective than Ca (HR = 0.78, 95% *CrI* = 0.65-0.94; HR = 0.68, 95% *CrI* = 0.52-0.88; HR = 0.76, 95% *CrI* = 0.59-0.97). When it came to 3-y PFS, D/Ca, Pa/Ca, Pa/E/Ca, PLD/Ca, PLD/Pa/Ca and T/Pa/Ca were preferred compared to Ca (HR = 0.82, 95% *CrI* = 0.68-0.99; HR = 0.84, 95% *CrI* = 0.76-0.94; HR = 0.80, 95% *CrI* = 0.67-0.96; HR = 0.75, 95% *CrI* = 0.65-0.86; HR = 0.83, 95% *CrI* = 0.69-0.99; HR = 0.87, 95% *CrI* = 0.76-0.99). In addition, PLD/Ca displayed stronger efficacy in reference to G/Ca, G/Pa/Ca and Pa/Ca respectively (HR = 0.80, 95% *CrI* = 0.65-0.99; HR = 0.83, 95% *CrI* = 0.72-0.95; HR = 0.88, 95% *CrI* = 0.80-0.98). While T/Pa/Ca appeared to be less favorable in the comparison with PLD/Ca (HR = 1.16, 95% *CrI* = 1.02-1.32). Similar results could be found according to 5y-PFS, showing that Pa/Ca and Pa/E/Ca were notably better than Ca (HR = 0.84, 95% *CrI* = 0.74-0.96; HR = 0.80, 95% *CrI* = 0.65-0.99).

**Table 2:** Network meta-analysis results of efficacy outcomes

1y-OS												
	Ca	Cy/D/Ci	D/Ca	G/Ca	G/Pa/Ca	Ia/Ca	Ir/Ci	Pa/Ca	Pa/E/Ca	PLD/Ca	PLD/Pa/Ca	T/Pa/Ca
Ca	1	0.67 (0.35, 1.26)	1.02 (0.75, 1.40)	0.99 (0.47, 2.08)	0.95 (0.73, 1.23)	1.05 (0.02, 51.38)	0.94 (0.24, 3.70)	0.94 (0.73, 1.21)	0.98 (0.59, 1.65)	0.94 (0.53, 1.68)	0.89 (0.66, 1.21)	0.98 (0.74, 1.29)
Cy/D/Ci	0.82 (0.54, 1.26)	1	1.54 (0.83, 2.84)	1.49 (0.60, 3.70)	1.42 (0.79, 2.56)	1.58 (0.03, 81.33)	1.41 (0.32, 6.14)	1.41 (0.78, 2.53)	1.48 (0.71, 3.09)	1.41 (0.64, 3.10)	1.34 (0.73, 2.46)	1.47 (0.81, 2.67)
D/Ca	0.83 (0.61, 1.12)	1.00 (0.64, 1.58)	1	0.97 (0.47, 1.99)	0.93 (0.76, 1.13)	1.03 (0.02, 50.93)	0.92 (0.23, 3.58)	0.92 (0.76, 1.10)	0.96 (0.59, 1.56)	0.92 (0.53, 1.61)	0.87 (0.68, 1.12)	0.96 (0.77, 1.19)
G/Ca	0.82 (0.55, 1.23)	1.00 (0.59, 1.69)	1.00 (0.65, 1.54)	1	0.95 (0.47, 1.91)	1.06 (0.02, 55.43)	0.94 (0.21, 4.30)	0.94 (0.47, 1.89)	0.99 (0.43, 2.26)	0.95 (0.40, 2.26)	0.90 (0.44, 1.83)	0.98 (0.49, 1.99)
G/Pa/Ca	0.79 (0.61, 1.01)	0.96 (0.63, 1.45)	0.95 (0.71, 1.28)	0.96 (0.64, 1.43)	1	1.11 (0.02, 54.76)	0.99 (0.26, 3.83)	0.99 (0.93, 1.06)	1.04 (0.66, 1.63)	0.99 (0.59, 1.69)	0.94 (0.79, 1.13)	1.03 (0.90, 1.18)
Ia/Ca	1.06 (0.49, 2.30)	1.29 (0.53, 3.12)	1.28 (0.56, 2.95)	1.29 (0.54, 3.09)	1.35 (0.60, 3.03)	1	0.89 (0.01, 55.29)	0.89 (0.02, 44.05)	0.94 (0.02, 47.46)	0.90 (0.02, 45.79)	0.85 (0.02, 42.0)	0.93 (0.02, 45.95)
Ir/Ci	0.80 (0.43, 1.49)	0.97 (0.48, 1.97)	0.97 (0.51, 1.83)	0.97 (0.49, 1.95)	1.01 (0.55, 1.88)	0.75 (0.28, 2.03)	1	1.00 (0.26, 3.86)	1.05 (0.25, 4.35)	1.00 (0.24, 4.27)	0.95 (0.24, 3.70)	1.04 (0.27, 4.04)
Pa/Ca	**0.78 (0.65, 0.94)**	0.95 (0.65, 1.39)	0.95 (0.75, 1.21)	0.95 (0.66, 1.37)	0.99 (0.84, 1.17)	0.74 (0.33, 1.63)	0.98 (0.54, 1.77)	1	1.05 (0.67, 1.64)	1.00 (0.59, 1.70)	0.95 (0.80, 1.12)	1.04 (0.92, 1.18)
Pa/E/Ca	0.78 (0.54, 1.13)	0.95 (0.58, 1.57)	0.95 (0.63, 1.42)	0.95 (0.59, 1.54)	0.99 (0.69, 1.43)	0.74 (0.31, 1.74)	0.98 (0.50, 1.92)	1.00 (0.73, 1.38)	1	0.96 (0.48, 1.91)	0.90 (0.56, 1.46)	0.99 (0.62, 1.58)
PLD/Ca	**0.68 (0.52, 0.88)**	0.82 (0.54, 1.26)	0.82 (0.60, 1.11)	0.82 (0.55, 1.24)	0.86 (0.67, 1.11)	0.64 (0.28, 1.44)	0.85 (0.45, 1.58)	0.86 (0.71, 1.05)	0.86 (0.59, 1.25)	1	0.95 (0.55, 1.64)	1.04 (0.60, 1.78)
PLD/Pa/Ca	0.77 (0.55, 1.06)	0.93 (0.59, 1.49)	0.93 (0.65, 1.33)	0.93 (0.60, 1.46)	0.97 (0.71, 1.34)	0.72 (0.31, 1.67)	0.96 (0.50, 1.84)	0.98 (0.75, 1.28)	0.98 (0.65, 1.49)	1.14 (0.82, 1.58)	1	1.10 (0.89, 1.35)
T/Pa/Ca	**0.76 (0.59, 0.97)**	0.92 (0.61, 1.39)	0.92 (0.69, 1.22)	0.92 (0.62, 1.37)	0.96 (0.76, 1.21)	0.71 (0.32, 1.61)	0.95 (0.51, 1.75)	0.97 (0.82, 1.14)	0.97 (0.67, 1.39)	1.12 (0.87, 1.44)	0.99 (0.72, 1.35)	1
1y-PFS												
3y-OS												
	Ca	Cy/D/Ci	D/Ca	G/Ca	G/Pa/Ca	Ia/Ca	Ir/Ci	Pa/Ca	Pa/E/Ca	PLD/Ca	PLD/Pa/Ca	T/Pa/Ca
Ca	1	0.81 (0.58, 1.12)	1.01 (0.79, 1.29)	1.07 (0.77, 1.49)	0.89 (0.76, 1.05)	1.23 (0.63, 2.41)	0.87 (0.52, 1.48)	0.89 (0.78, 1.02)	0.90 (0.70, 1.16)	0.90 (0.69, 1.16)	0.85 (0.68, 1.05)	0.92 (0.77, 1.10)
Cy/D/Ci	0.89 (0.70, 1.13)	1	1.24 (0.87, 1.78)	1.32 (0.87, 2.01)	1.10 (0.81, 1.50)	1.52 (0.72, 3.20)	1.08 (0.60, 1.94)	1.10 (0.82, 1.48)	1.11 (0.77, 1.60)	1.10 (0.76, 1.60)	1.04 (0.74, 1.47)	1.13 (0.83, 1.56)
D/Ca	**0.82 (0.68, 0.99)**	0.92 (0.71, 1.21)	1	1.06 (0.74, 1.53)	0.89 (0.71, 1.11)	1.22 (0.60, 2.50)	0.87 (0.50, 1.50)	0.88 (0.72, 1.09)	0.89 (0.66, 1.20)	0.89 (0.65, 1.21)	0.84 (0.64, 1.09)	0.91 (0.72, 1.15)
G/Ca	0.93 (0.75, 1.15)	1.05 (0.79, 1.40)	1.13 (0.89, 1.45)	1	0.84 (0.61, 1.14)	1.15 (0.55, 2.43)	0.82 (0.45, 1.47)	0.83 (0.62, 1.12)	0.84 (0.58, 1.21)	0.84 (0.58, 1.22)	0.79 (0.56, 1.11)	0.86 (0.62, 1.18)
G/Pa/Ca	0.90 (0.79, 1.04)	1.02 (0.81, 1.29)	1.10 (0.92, 1.32)	0.97 (0.79, 1.20)	1	1.38 (0.69, 2.74)	0.98 (0.58, 1.64)	1.00 (0.91, 1.09)	1.01 (0.80, 1.26)	1.00 (0.79, 1.28)	0.95 (0.78, 1.14)	1.03 (0.89, 1.18)
Ia/Ca	1.19 (0.72, 1.98)	1.34 (0.76, 2.35)	1.45 (0.84, 2.49)	1.28 (0.74, 2.23)	1.32 (0.78, 2.23)	1	0.71 (0.30, 1.66)	0.72 (0.37, 1.44)	0.73 (0.36, 1.50)	0.73 (0.35, 1.50)	0.69 (0.34, 1.39)	0.75 (0.37, 1.49)
Ir/Ci	0.95 (0.61, 1.48)	1.08 (0.67, 1.74)	1.16 (0.74, 1.84)	1.03 (0.64, 1.64)	1.06 (0.68, 1.64)	0.80 (0.41, 1.57)	1	1.02 (0.61, 1.70)	1.03 (0.59, 1.79)	1.03 (0.59, 1.79)	0.97 (0.57, 1.65)	1.05 (0.63, 1.77)
Pa/Ca	**0.84 (0.76, 0.94)**	0.95 (0.77, 1.18)	1.03 (0.88, 1.20)	0.91 (0.75, 1.10)	0.93 (0.85, 1.02)	0.71 (0.42, 1.19)	0.88 (0.58, 1.36)	1	1.01 (0.82, 1.25)	1.01 (0.80, 1.26)	0.95 (0.80, 1.12)	1.03 (0.92, 1.15)
Pa/E/Ca	**0.80 (0.67, 0.96)**	0.90 (0.70, 1.18)	0.98 (0.79, 1.21)	0.86 (0.68, 1.10)	0.89 (0.75, 1.06)	0.67 (0.39, 1.16)	0.84 (0.53, 1.32)	0.95 (0.82, 1.10)	1	1.00 (0.73, 1.36)	0.94 (0.72, 1.23)	1.02 (0.80, 1.30)
PLD/Ca	**0.75 (0.65, 0.86)**	0.84 (0.66, 1.07)	0.91 (0.76, 1.09)	**0.80 (0.65, 0.99)**	**0.83 (0.72, 0.95)**	0.63 (0.37, 1.06)	0.78 (0.50, 1.22)	**0.88 (0.80, 0.98)**	0.93 (0.78, 1.11)	1	0.94 (0.71, 1.25)	1.03 (0.80, 1.32)
PLD/Pa/Ca	**0.83 (0.69, 0.99)**	0.93 (0.72, 1.21)	1.01 (0.82, 1.25)	0.89 (0.70, 1.13)	0.92 (0.77, 1.08)	0.70 (0.41, 1.19)	0.87 (0.55, 1.36)	0.98 (0.85, 1.13)	1.03 (0.84, 1.27)	1.11 (0.93, 1.32)	1	1.09 (0.89, 1.33)
T/Pa/Ca	**0.87 (0.76, 0.99)**	0.98 (0.77, 1.24)	1.06 (0.89, 1.26)	0.93 (0.76, 1.15)	0.96 (0.85, 1.09)	0.73 (0.43, 1.23)	0.91 (0.59, 1.41)	1.03 (0.94, 1.12)	1.08 (0.91, 1.28)	**1.16 (1.02, 1.32)**	1.05 (0.89, 1.24)	1
3y-PFS												
5y-OS												
	Ca	Cy/D/Ci	G/Ca	G/Pa/Ca	Ia/Ca	Ir/Ci	Pa/Ca	Pa/E/Ca	PLD/Ca	PLD/Pa/Ca	T/Pa/Ca	
Ca	1	0.86 (0.59, 1.24)	1.10 (0.76, 1.61)	0.86 (0.59, 1.25)	1.17 (0.66, 2.07)	0.96 (0.60, 1.53)	0.85 (0.70, 1.03)	0.79 (0.56, 1.11)	0.86 (0.64, 1.16)	0.81 (0.55, 1.19)	0.84 (0.65, 1.10)	
Cy/D/Ci	0.89 (0.68, 1.15)	1	1.29 (0.82, 2.01)	1.00 (0.64, 1.57)	1.36 (0.69, 2.68)	1.12 (0.66, 1.90)	0.99 (0.73, 1.35)	0.92 (0.61, 1.40)	1.01 (0.69, 1.48)	0.94 (0.60, 1.48)	0.98 (0.68, 1.41)	
G/Ca	0.94 (0.74, 1.19)	1.06 (0.78, 1.43)	1	0.78 (0.49, 1.23)	1.06 (0.54, 2.09)	0.87 (0.51, 1.48)	0.77 (0.56, 1.06)	0.72 (0.47, 1.09)	0.78 (0.53, 1.16)	0.73 (0.46, 1.16)	0.76 (0.53, 1.10)	
G/Pa/Ca	0.94 (0.79, 1.12)	1.06 (0.82, 1.37)	1.01 (0.79, 1.28)	1	1.36 (0.69, 2.70)	1.12 (0.65, 1.91)	0.99 (0.72, 1.37)	0.92 (0.60, 1.41)	1.01 (0.68, 1.50)	0.94 (0.59, 1.50)	0.98 (0.68, 1.42)	
Ia/Ca	1.13 (0.73, 1.75)	1.28 (0.77, 2.12)	1.21 (0.73, 1.99)	1.20 (0.75, 1.92)	1	0.82 (0.39, 1.71)	0.73 (0.40, 1.32)	0.68 (0.35, 1.31)	0.74 (0.39, 1.40)	0.69 (0.35, 1.37)	0.72 (0.38, 1.35)	
Ir/Ci	0.99 (0.70, 1.39)	1.11 (0.75, 1.65)	1.05 (0.72, 1.54)	1.05 (0.74, 1.48)	0.87 (0.50, 1.52)	1	0.88 (0.58, 1.36)	0.82 (0.49, 1.37)	0.90 (0.56, 1.46)	0.84 (0.49, 1.44)	0.88 (0.55, 1.39)	
Pa/Ca	**0.84 (0.74, 0.96)**	0.95 (0.76, 1.19)	0.90 (0.73, 1.11)	0.90 (0.79, 1.01)	0.75 (0.47, 1.18)	0.85 (0.62, 1.18)	1	0.93 (0.71, 1.23)	1.02 (0.81, 1.27)	0.95 (0.68, 1.33)	0.99 (0.83, 1.19)	
Pa/E/Ca	**0.80 (0.65, 0.99)**	0.90 (0.68, 1.20)	0.86 (0.65, 1.12)	0.85 (0.69, 1.05)	0.71 (0.44, 1.15)	0.81 (0.56, 1.17)	0.95 (0.80, 1.13)	1	1.09 (0.77, 1.56)	1.02 (0.66, 1.57)	1.07 (0.77, 1.48)	
PLD/Ca	0.81 (0.66, 1.01)	0.92 (0.69, 1.22)	0.87 (0.66, 1.14)	0.86 (0.70, 1.07)	0.72 (0.44, 1.17)	0.82 (0.57, 1.19)	0.97 (0.81, 1.15)	1.02 (0.80, 1.30)	1	0.93 (0.62, 1.39)	0.97 (0.73, 1.30)	
PLD/Pa/Ca	0.83 (0.65, 1.05)	0.93 (0.69, 1.26)	0.88 (0.66, 1.18)	0.88 (0.69, 1.11)	0.73 (0.44, 1.20)	0.84 (0.57, 1.22)	0.98 (0.80, 1.20)	1.03 (0.79, 1.34)	1.02 (0.78, 1.32)	1	1.04 (0.71, 1.52)	
T/Pa/Ca	0.87 (0.74, 1.03)	0.98 (0.77, 1.27)	0.93 (0.74, 1.18)	0.93 (0.79, 1.09)	0.77 (0.48, 1.23)	0.88 (0.63, 1.24)	1.03 (0.93, 1.15)	1.09 (0.89, 1.34)	1.07 (0.87, 1.32)	1.06 (0.84, 1.33)	1	
5y-PFS												

Note: Hazard ratio (HR) and corresponding 95% *CrI* for efficacy outcomes. In the upper regions, columns are compared with rows while lower regions are opposite. Abbreviations: OS: Overall survival; PFS: Progression-free survival; Ir: Irinotecan; Ci: Cisplatin; Pa: Paclitaxel; Ca: Carboplatin; PLD: Pegylated liposomal doxorubicin; G: Gemcitabine; T: Topotecan; D: Doxorubicin; Cy: Cyclophosphamide; Ia: Interferon-alpha; E: Epirubicin. Boldfaced nunbers indicate significance difference.

**Figure 3:** Forest plot of the efficacy outcomes Results are expressed as hazard ratio (HR) with 95% credible interval (CrI). Abbreviation: OS: Overall survival; PFS: Progression-free survival; Ir: Irinotecan; Ci: Cisplatin; Pa: Paclitaxel; Ca: Carboplatin; PLD: Pegylated liposomal doxorubicin; G: Gemcitabine; T: Topotecan; D: Doxorubicin; Cy: Cyclophosphamide; Ia: Interferon-alpha; E: Epirubicin.

In adverse effect analysis, 6 different outcomes were measured. Alopecia was included in 13 trials, while neutropenia, nausea, vomiting, diarrhea and neuropathy were recorded in 10, 12, 16, 11 and 16 trials respectively. In Table 3 all direct comparisons and indirect comparisons were measured with OR of each adverse effect. As a wide-used therapy, Ca significantly decreased the occurrence of neutropenia compared to other therapies such as D/Ca, G/Ca, G/Pa/Ca, Ir/Ci, Pa/Ca, PLD/Ca and T/Pa/Ca. On the other hand, T/Pa/Ca showed inferior position compared with G/Ca, Ir/Ci, Pa/Ca and PLD/Ca. As for neuropathy, patients treated with Ca exhibited a reduced risk compared to D/Ca, G/Pa/Ca, Pa/Ca, Pa/E/Ca, PLD/Ca and T/Pa/Ca. Cy/D/Ci significantly decreased the risk in comparison with G/Pa/Ca, Pa/Ca, Pa/E/Ca and T/Pa/Ca. G/Ca shared the same characteristic as Cy/D/Ci. D/Ca performed worse compared to G/Ca, Ia/Ca, Ir/Ci and PLD/Ca. Besides, G/Pa/Ca was also inferior to Ia/Ca, Ir/Ci and PLD/Ca. Patients treated by Ia/Ca exhibited lower neuropathy risk compared to Pa/Ca, Pa/E/Ca and T/Pa/Ca. Ir/Ci was notably better than Pa/Ca, Pa/E/Ca, PLD/Ca and T/Pa/Ca. Additionally, PLD/Ca was preferred compared to Pa/Ca and Pa/E/Ca while it was superior compared to T/Pa/Ca. Patients with Ir/Ci exhibited an increased risk of diarrhea compared to Pa/Ca, Pa/E/Ca, PLD/Ca, T/Pa/Ca and G/Pa/Ca. As to Alopecia, Ca showed better safety compared to Cy/D/Ci, G/Pa/Ca, Pa/Ca and T/Pa/Ca. Ir/Ci was preferred compared to Cy/D/Ci, G/Pa/Ca, Pa/Ca and T/Pa/Ca. Besides, PLD/Ca was superior to Cy/D/Ci, G/Pa/Ca, Pa/Ca and T/Pa/Ca. With respect to nausea, only Pa/Ca demonstrated less effect than Ir/Ci. In addition, patients treated by Ir/Ci exhibited more vomiting compared to Ca, D/Ca, G/Ca, G/Pa/Ca, Pa/Ca and PLD/Ca. Patients in Cy/D/Ci treatment exhibited more vomiting side effect compared to Pa/Ca and G/Pa/Ca.

**Table 3:** Network meta-analysis results of adverse effects

Neutropenia											
	Ca	Cy/D/Ci	D/Ca	G/Ca	G/Pa/Ca	Ia/Ca	Ir/Ci	Pa/Ca	Pa/E/Ca	PLD/Ca	T/Pa/Ca
Ca	1	-	**69.41 (3.22, 2440.6)**	**14.44 (2.39, 165.7)**	**24.78 (4.22, 275.9)**	**-**	**8.41 (1.27, 105.6)**	**12.81 (2.41, 126.5)**	**-**	**15.33 (2.97, 144.0)**	**66.69 (9.39, 804.3)**
Cy/D/Ci	0.3 (0.08, 1.27)	1	-	-	-	-	-	-	-	-	-
D/Ca	**0.09 (0.03, 0.31)**	0.29 (0.08, 1.06)	1	0.22 (0.01, 2.69)	0.36 (0.02, 4.48)	-	0.13 (0.01, 1.70)	0.2 (0.01, 2.14)	-	0.23 (0.02, 2.61)	1.02 (0.06, 13.2)
G/Ca	0.36 (0.10, 1.55)	1.19 (0.27, 5.53)	**4.06 (1.08, 15.49)**	1	1.7 (0.63, 4.48)	-	0.59 (0.18, 1.77)	0.89 (0.44, 1.79)	-	1.06 (0.47, 2.32)	**4.53 (1.43, 15.0)**
G/Pa/Ca	**0.05 (0.02, 0.18)**	**0.16 (0.04, 0.62)**	0.55 (0.17, 1.73)	**0.14 (0.03, 0.52)**	1	-	0.35 (0.11, 1.06)	0.52 (0.26, 1.05)	-	0.63 (0.28, 1.35)	2.69 (0.85, 8.67)
Ia/Ca	1.38 (0.27, 7.61)	4.57 (0.53, 37.71)	**15.49 (2.03, 120.3)**	3.82 (0.43, 32.46)	**28.22 (3.53, 223.63)**	1	-	-	-	-	-
Ir/Ci	1.14 (0.34, 4.39)	3.74 (0.93, 15.18)	**12.94 (3.86, 42.52)**	3.19 (0.76, 12.94)	**23.57 (6.62, 83.1)**	0.84 (0.10, 6.82)	1	1.49 (0.61, 3.86)	-	1.8 (0.68, 4.95)	**7.69 (2.16, 29.9)**
Pa/Ca	**0.05 (0.02, 0.12)**	**0.16 (0.05, 0.44)**	0.54 (0.24, 1.16)	**0.13 (0.04, 0.38)**	0.98 (0.41, 2.32)	**0.03 (0.01, 0.23)**	**0.04 (0.02, 0.1)**	1	-	1.21 (0.82, 1.72)	**5.05 (2.05, 13.6)**
Pa/E/Ca	**0.05 (0.02, 0.19)**	**0.17 (0.04, 0.66)**	0.59 (0.18, 1.86)	**0.15 (0.04, 0.57)**	1.08 (0.32, 3.63)	**0.04 (0.01, 0.31)**	**0.05 (0.01, 0.16)**	1.09 (0.46, 2.56)	1	-	**-**
PLD/Ca	**0.24 (0.09, 0.72)**	0.77 (0.25, 2.56)	**2.64 (1.13, 6.96)**	0.66 (0.21, 2.23)	**4.76 (1.95, 13.74)**	0.17 (0.03, 1.27)	**0.20 (0.08, 0.61)**	**4.90 (3.22, 8.58)**	**4.44 (1.80, 12.94)**	1	**4.22 (1.62, 12.3)**
T/Pa/Ca	**0.04 (0.02, 0.14)**	**0.15 (0.04, 0.49)**	0.50 (0.18, 1.34)	**0.12 (0.03, 0.42)**	0.90 (0.30, 2.66)	**0.03 (0.01, 0.24)**	**0.04 (0.01, 0.12)**	0.92 (0.47, 1.77)	0.84 (0.28, 2.48)	**0.19 (0.08, 0.39)**	1
**Neuropathy**											
**Diarrhea**											
	Ca	Cy/D/Ci	D/Ca	G/Ca	G/Pa/Ca	Ia/Ca	Ir/Ci	Pa/Ca	Pa/E/Ca	PLD/Ca	T/Pa/Ca
Ca	1	-	0.62 (0.05, 6.23)	-	0.61 (0.05, 5.93)	0.93 (0.07, 12.94)	4.31 (0.36, 42.52)	0.45 (0.06, 2.97)	0.56 (0.05, 5.53)	0.26 (0.03, 2.01)	0.49 (0.04, 5.26)
Cy/D/Ci	**0.05 (0.01, 0.57)**	1	-	-	-	-	-	-	-	-	-
D/Ca	**-**	-	1	-	0.98 (0.14, 6.82)	1.55 (0.05, 55.15)	7.03 (0.98, 48.91)	0.73 (0.18, 2.97)	0.91 (0.14, 6.36)	0.42 (0.09, 2.10)	0.79 (0.11, 5.99)
G/Ca	0.50 (0.04, 6.30)	10.8 (0.52, 230.44)	-	1	-	-	-	-	-	-	-
G/Pa/Ca	**0.06 (0.01, 0.72)**	1.27 (0.06, 26.31)	-	0.12 (0.01, 2.51)	1	1.57 (0.05, 52.98)	**7.10 (1.05, 46.99)**	0.74 (0.19, 2.83)	0.93 (0.14, 6.30)	0.44 (0.09, 1.99)	0.82 (0.11, 5.87)
Ia/Ca	0.99 (0.10, 9.49)	21.54 (0.69, 626.41)	-	1.97 (0.07, 57.4)	16.95 (0.57, 497.7)	1	4.57 (0.13, 145.47)	0.47 (0.02, 12.06)	0.59 (0.02, 18.92)	0.28 (0.01, 7.32)	0.51 (0.01, 16.78)
Ir/Ci	4.26 (0.20, 239.85)	**93.69 (2.83, 7331.97)**	-	8.67 (0.25, 678.58)	**73.7 (2.18, 5825.5)**	4.44 (0.09, 432.68)	1	**0.10 (0.03, 0.41)**	**0.13 (0.02, 0.91)**	**0.06 (0.01, 0.30)**	**0.11 (0.02, 0.83)**
Pa/Ca	**0.04 (0.01, 0.14)**	0.82 (0.09, 6.96)	-	**0.08 (0.01, 0.64)**	0.64 (0.07, 5.53)	**0.04 (0.01, 0.53)**	**0.01 (0.01, 0.14)**	1	1.26 (0.33, 4.90)	0.58 (0.28, 1.22)	1.11 (0.26, 4.62)
Pa/E/Ca	-	-	-	-	-	-	-	-	1	0.46 (0.10, 2.14)	0.88 (0.12, 6.11)
PLD/Ca	0.75 (0.14, 4.22)	**16.28 (1.54, 186.79)**	-	1.49 (0.14, 16.95)	**12.68 (1.17, 149.9)**	0.76 (0.05, 13.33)	0.18 (0.01, 3.60)	**19.89 (6.89, 61.56)**	-	1	1.90 (0.37, 9.30)
T/Pa/Ca	**0.03 (0.01, 0.37)**	0.66 (0.03, 13.87)	-	0.06 (0.01, 1.25)	0.52 (0.02, 10.8)	**0.03 (0.01, 0.89)**	**0.01 (0.01, 0.23)**	0.81 (0.09, 6.89)	-	**0.04 (0.01, 0.44)**	1
**Alopecia**											
**Nausea**											
	Ca	Cy/D/Ci	D/Ca	G/Ca	G/Pa/Ca	Ir/Ci	Pa/Ca	Pa/E/Ca	PLD/Ca	T/Pa/Ca	
Ca	1	-	1.12 (0.29, 4.66)	0.78 (0.19, 3.63)	0.74 (0.20, 3.03)	2.41 (0.63, 10.28)	0.66 (0.23, 2.01)	1.21 (0.32, 4.95)	0.98 (0.33, 3.29)	0.85 (0.24, 3.16)	
Cy/D/Ci	0.45 (0.18, 1.15)	1	-	-	-	-	-	-	-	-	
D/Ca	1.55 (0.66, 3.78)	3.46 (1.15, 10.28)	1	0.7 (0.19, 2.66)	0.66 (0.20, 2.29)	2.14 (0.61, 7.69)	0.59 (0.24, 1.43)	1.07 (0.31, 3.78)	0.86 (0.34, 2.56)	0.76 (0.25, 2.29)	
G/Ca	1.23 (0.45, 3.49)	2.75 (0.81, 9.30)	0.79 (0.24, 2.61)	1	0.96 (0.26, 3.53)	3.10 (0.79, 12.06)	0.85 (0.30, 2.32)	1.55 (0.41, 5.81)	1.25 (0.42, 4.06)	1.09 (0.32, 3.63)	
G/Pa/Ca	1.36 (0.63, 3.06)	**3.03 (1.08, 8.50)**	0.88 (0.32, 2.36)	1.11 (0.36, 3.39)	1	3.22 (0.94, 11.36)	0.89 (0.38, 2.08)	1.62 (0.49, 5.42)	1.30 (0.53, 3.74)	1.14 (0.39, 3.32)	
Ir/Ci	**0.34 (0.15, 0.79)**	0.76 (0.26, 2.18)	**0.22 (0.08, 0.61)**	**0.28 (0.09, 0.87)**	**0.25 (0.10, 0.64)**	1	**0.28 (0.11, 0.68)**	0.51 (0.14, 1.75)	0.41 (0.15, 1.20)	0.35 (0.11, 1.07)	
Pa/Ca	1.16 (0.76, 1.84)	**2.56 (1.16, 5.75)**	0.75 (0.35, 1.58)	0.94 (0.38, 2.36)	0.85 (0.44, 1.63)	**3.39 (1.70, 6.82)**	1	1.82 (0.77, 4.35)	1.46 (0.95, 2.61)	1.28 (0.65, 2.51)	
Pa/E/Ca	0.73 (0.34, 1.67)	1.62 (0.58, 4.57)	0.47 (0.18, 1.27)	0.59 (0.19, 1.80)	0.53 (0.21, 1.36)	2.14 (0.83, 5.64)	0.63 (0.33, 1.22)	1	0.79 (0.31, 2.34)	0.70 (0.23, 2.05)	
PLD/Ca	0.88 (0.51, 1.60)	1.95 (0.81, 4.76)	0.57 (0.25, 1.31)	0.71 (0.27, 1.93)	0.64 (0.31, 1.38)	**2.56 (1.19, 5.75)**	0.76 (0.53, 1.11)	1.20 (0.57, 2.56)	1	0.88 (0.35, 1.90)	
T/Pa/Ca	0.67 (0.31, 1.48)	1.48 (0.54, 4.22)	0.43 (0.16, 1.15)	0.54 (0.18, 1.65)	0.49 (0.20, 1.21)	1.95 (0.77, 5.00)	0.58 (0.30, 1.08)	0.92 (0.37, 2.27)	0.76 (0.36, 1.57)	1	
**Vomiting**											

Note: Odds ratio (OR) and corresponding 95% *CrI* for safety outcomes. In the upper regions, columns are compared with rows while lower regions are opposite. Abbreviations: Ir: Irinotecan; Ci: Cisplatin; Pa: Paclitaxel; Ca: Carboplatin; PLD: Pegylated liposomal doxorubicin; G: Gemcitabine; T: Topotecan; D: Doxorubicin; Cy: Cyclophosphamide; Ia: Interferon-alpha; E: Epirubicin. Boldfaced nunbers indicate significance difference.

### Ranking of therapies

To determine which therapy could be the best, SUCRA was introduced to show the ranking of each treatment (Table 4). According to the results, Cy/D/Ci performed well in survival measurements (1y-OS: SUCRA 0.819; 3y-OS: SUCRA 0.763), while PLD/Ca exhibited the best efficacy in 1y-PFS (SUCRA 0.844) and 3y-PFS (SUCRA 0.927). PLD/Pa/Ca achieved upper class rankings in all outcomes measurements (1y-OS: SUCRA 0.637; 1y-PFS: SUCRA 0.592; 3y-OS: SUCRA 0.737; 3y-PFS: SUCRA 0.663; 5y-OS: SUCRA 0.687; 5y-PFS: SUCRA 0.712). In addition, Pa/E/Ca and PLD/Ca were top two in 5y-PFS (SUCRA 0.798; SUCRA 0.759). The rankings of different therapies were illustrated in a cluster plot where each part contained a pair of measurements and the upper right area meant a higher ranking in these two measurements. According to Figure 4, PLD/Pa/Ca ranked the best regarding 3y-PFS & 3y-OS and 5y-PFS & 3y-OS. Also, the results showed that Pa/E/Ca was in the first class considering 3y-PFS & 5y-OS and 5y-PFS & 5y-OS. As for side effect, Ca appeared to have much less possibility of causing neutropenia, neuropathy and alopecia. Ia/Ca and Ir/Ci were superior in avoiding neuropathy and alopecia than other interventions. Pa/Ca was relatively safer in causing neutropenia, diarrhea, nausea and vomiting, while PLD/Ca ranked the first with respect to diarrhea, indicating its low risk of making patients experience diarrhea.

**Table 4:** SUCRA of different outcomes

Treatments	Primary outcomes						Adverse effects					
	1y-OS	1y-PFS	3y-OS	3y-PFS	5y-OS	5y-PFS	Neutropenia	Neuropathy	Diarrhea	Alopecia	Nausea	Vomiting
**Ca**	**0.394**	**0.133**	**0.282**	**0.157**	**0.280**	**0.207**	**0.996**	**0.862**	**0.471**	**0.757**	**0.484**	**0.577**
Cy/D/Ci	**0.819**	0.470	**0.763**	0.467	0.583	0.531	-	0.618	-	0.222	-	0.141
D/Ca	0.334	0.444	0.297	**0.687**	-	-	0.159	0.376	0.601	-	0.380	**0.865**
G/Ca	0.445	0.468	0.235	0.343	0.184	0.387	0.546	0.657	-	0.603	**0.653**	0.713
G/Pa/Ca	0.499	0.538	0.601	0.374	0.582	0.345	0.280	0.168	0.603	0.270	**0.704**	**0.811**
Ia/Ca	0.476	0.260	0.216	0.139	0.214	0.177	-	**0.899**	0.523	**0.735**	-	-
Ir/Ci	0.499	0.518	0.591	0.371	0.405	0.316	-	**0.893**	0.172	**0.923**	0.051	0.049
Pa/Ca	**0.540**	0.549	**0.622**	0.616	0.622	0.696	**0.789**	0.152	**0.806**	0.166	**0.846**	**0.721**
Pa/E/Ca	0.441	0.551	0.570	**0.749**	**0.738**	**0.798**	**0.661**	0.208	0.647	-	0.318	0.350
PLD/Ca	0.499	**0.844**	0.579	**0.927**	0.572	**0.759**	0.489	0.553	**0.961**	0.684	0.470	0.467
PLD/Pa/Ca	**0.637**	**0.592**	**0.737**	0.663	**0.687**	**0.712**	-	-	-	-	-	-
T/Pa/Ca	0.417	0.633	0.507	0.509	**0.634**	0.572	0.080	0.113	**0.715**	0.140	0.594	0.307

Abbreviations: OS: Overall survival; PFS: Progression-free survival; Ir: Irinotecan; Ci: Cisplatin; Pa: Paclitaxel; Ca: Carboplatin; PLD: Pegylated liposomal doxorubicin; G: Gemcitabine; T: Topotecan; D: Doxorubicin; Cy: Cyclophosphamide; Ia: Interferon-alpha; E: Epirubicin. The warmer the color of the cell is, the higher the corresponding intervention ranks under the related outcome. Boldfaced numbers indicate the top three rankings for each outcome.

**Figure 4:** Cluster analysis of long-term efficacy outcomes Treatments in orange suggest a high ranking in both horizontal and vertical ordinate outcomes and treatments in blue suggest a low ranking. Abbreviation: OS: Overall survival; PFS: Progression-free survival; Ir: Irinotecan; Ci: Cisplatin; Pa: Paclitaxel; Ca: Carboplatin; PLD: Pegylated liposomal doxorubicin; G: Gemcitabine; T: Topotecan; D: Doxorubicin; Cy: Cyclophosphamide; Ia: Interferon-alpha; E: Epirubicin.

## DISCUSSION

Ovarian cancer drew many people's attention all around the world as a highly risky cancer. In recent years, more and more papers are published to assess the efficacy and safety of different therapies for patients with ovarian cancer. Based on these RCTs and meta-analysis (MA) studies, our NMA study collected all available data and integrated the pair-wise comparisons into a network comparison from which we could interpret to find superior therapies. Although one NMA study has already been published, the shortage of this NMA study is that it did not the adverse effects into account. For instance, in this study [16] the author only considered the outcomes concerning efficacy like progressive disease and disease control rate and no effort was made to measure the toxicity of different therapies, which diluted its reference significance. Furthermore, the author failed to measure the effect of follow-up time by using HR to evaluate the survival outcome at different time point. Therefore our study has its necessity and accuracy in addressing these unresolved problems.

In the NMA study, six outcomes concerning efficacy and six outcomes concerning safety are collected and measured. According to the cluster plots and other measurements, PLD/Pa/Ca, PLD/Ca and Pa/E/Ca are highly recommended while G/Ca and Ia/Ca are regarded as worst therapies considering long-term OS and PFS. Although in none of these outcomes ranked first, the overall performance of PLD/Pa/Ca was better than other therapies with all outcomes above 0.5 and showed a potential of increasing along with the follow-up time. Studies [27, 28] showed that PLD /Ca or other therapies were more effective and the mechanism of PLD was thought to be able to reduce the synthesis of proteins, DNA and RNA [29]. That may be why the therapies including PLD proved to be effective in our study. On the other hand, Pa/E/Ca displayed better results in longer follow up time outcomes, compared with 1y-OS and 1y-PFS. In contrast, G/Ca and Ia/Ca performed badly in all primary outcomes, showing a decrease in ranking as the follow up time grew. Pa/Ca, as a basic treatment for ovarian cancer, performed a moderate ranking probability in all outcomes with second class efficacy in cluster analysis, which suggested that the use of Paclitaxel and Carboplatin with or without other combined chemical regimens might exhibit favorable efficacy, provided a rational strategy for later treatment design.

When it comes to adverse effects, neutropenia and neuropathy were considered as the primary outcomes among all the adverse effects caused by chemo treatments for ovarian cancer, and no further conclusion could be made because the measurements regarding several treatments were missing. Still, the results of adverse effects can serve as an aid to the drug ranking, considering Pa/E/Ca performed well in neutropenia but badly in neuropathy while G/Ca and PLD/Ca performed was surprisingly well. The transformation of doxorubicin in PLD increases the time the drug's circulating half-life, thus decreasing its toxicity [30]. Moreover, one study [31] illustrated that G/Ca was superior to those Pa/Ca based therapies, which was consistent with our findings. Due to the potential side effects, doctors should prescribe those treatments of high efficacy but serious adverse effects with caution, depending on the severity of condition and patients’ tolerance of adverse effects.

Besides, some interesting points remained to be discussed. First, it seemed that therapies with high rankings of safety inversely showed bad performance in rankings of efficacy. Ca was such a typical example that on the one hand it showed the highest rankings in safety while on the other hand its primary outcomes concerning efficacy was the worst. Similarly, Ia/Ca, G/Ca and other low efficacy ranking therapies all performed well in adverse effects. Second, the combinations of three compounds suggested better responses compared with the combinations of two compounds. Cy/D/Ci, Pa/E/Ca, Pa/E/Ca and PLD/Pa/Ca were located on the upper right area of the cluster plot, except G/Pa/Ca and T/Pa/Ca, while compared with Pa/Ca, Pa/E/Ca showed a better overall outcome of efficacy. Moreover, similar conclusions were offered that combination-platinum improved the primary outcomes [32]. However, further studies should be done on whether the number of compounds combined affecting the regimen's efficacy and safety as well.

Although this study was conducted as meticulous as possible, it still had limitations. Firstly, most of the RCTs involved in this study compared therapies with Pa/Ca, making the direct evidence between any other two treatments lacking, thus we could not get a further understanding in the inconsistency among these RCTs. Second, the primary outcomes of less recommended therapies were derived from a smaller sample size compared with recommended therapies, making the associated 95% *CrI* relatively greater and lowering the validity of results. It should be noted that the the significant difference of OS and PFS between comparisons as indicated by HR and 95% *CrI* had an upper limit approaching 1, which also weakened the credibility of the difference. Adverse effects, especially Alopecia, showed wide 95% *CrI* related to the ORs of different comparisons, the cause of which remained unclear. In addition, we could not find the adverse effects outcomes of PLD/Pa/Ca, though it was regarded as one of the recommended highly efficacious therapies among all therapies. Moreover, the different drug dose and patients’ physical condition in different researches were not mentioned in this study. As the number of included studies was limited, the differential analysis about the drug dose for each treatment could not be conducted. Similarly, an analysis about patients’ physical condition was not made, either, although the ovarian neoplasm tumors had different stages. Therefore, the suggestions made in this NMA should be adopted with reservation and more relevant large-sample studies that are focused on both efficacy and safety of various intervention comparisons for ovarian cancer should be conducted.

## CONCLUSIONS

In conclusion, PLD/Pa/Ca, PLD/Ca and Pa/E/Ca were highly recommended as potential choice of therapies for patients with ovarian cancer. But considering the lack of safety data for PLD/Pa/Ca, this intervention should be taken with caution. Still, the relationship between number of compounds in combination chemotherapies regarding both efficacy and safety remained to be figured out.

## MATERIALS AND METHODS

### Search strategy

Electronic databases such as PubMed, EMBASE were utilized to identify relevant trials. Besides, some other trial sources were utilized to ensure a comprehensive search result. To do the search, “ovarian neoplasms” and its subordinate entry terms were designated as keywords in title or abstract, while typical therapy terms were included in the strategies of searching in an “OR” form: “paclitaxel” (Pa), “carboplatin” (Ca), “gemcitabine” (G), “doxorubicin” (D), “pegylated liposomal doxorubicin” (PLD), “topotecan” (T), “epirubicin” (E), “interferon” (Ia) or “cyclophosphamide” (Cy). Further exclusion was made based on whether the study type was randomized controlled trials (RCTs).

### Selection criteria

For the NMA, all RCTs evaluating the efficacy and safety of drug therapies for ovarian neoplasm and including at least one pair of direct control group were potentially eligible. Furthermore, many trials were excluded for the following reasons: (1) duplicates; (2) articles based on the same clinical trials; (3) RCTs could not form a network; (4) data was insufficient or unavailable.

### Data extraction

Data extraction of characteristics and data from the included trials was accomplished independently by two reviewers. The following characteristics were included and collected: (1) study characteristics (author, publication year and country); (2) trial design characteristics (follow-up, sample size and comparison between therapies); (3) primary outcomes concerning efficacy (one year overall survival (1y-OS), 3y-OS, 5y-OS, One year progression-free survival (1y-PFS), 3y-PFS and 5y-PFS); (4) secondary outcome concerning safety and adverse effects (alopecia, neutropenia, nausea, vomiting, diarrhea and neuropathy). In fact, although complete response (CR) and partial response (PR) were equally vital in outcome measurements, they were excluded from data extracting because of a large number of missing information in included trials. Besides, neutropenia and neuropathy were considered as particularly important, compared with other adverse effects for severe damage against healthy.

### Statistical analysis

. R 3.3.2 and STATA 13.1 were applied to conduct the Bayesian NMA, and 95% *CrI* were computed for HR and OR in survival and adverse effect analysis.

For survival analysis, hazard ratio (HR) and the associated 95% credible interval (*CrI*) were used to describe efficacy in a comparison under OS and PFS measurements, and the results were presented as forest plots and relative effect tables. OS and PFS data of 3 year3y-OS, 5y-OS, 3y-PFS and 5y-PFS and 5 year were analyzed in a cluster plot, the treatments in the up-right corner indicated better efficacy.

For safety analysis, odds ratio (OR) and corresponding 95% *CrI* of each adverse effect were calculated. The different incidence rate of side effect (neutropenia, neuropathy, diarrhea, alopecia, nausea, vomiting) after medication was compared by relative OR and SUCRA value. Surface under the cumulative ranking curve (SUCRA) was calculated under each survival and safety outcome in order to compare the relative ranking of different therapies. A warmer color showed a higher rank in SUCRA table. R 3.3.2 and STATA 13.1 were applied to conduct the Bayesian NMA, and 95% *CrI* were computed for HR and OR in survival and adverse effect analysis.

Gongliang Guo designed the data collection instruments, carried out the initial analyses and approved the final manuscript as submitted.

Liqun Sun collected the data, carried out the initial analyses and approved the final manuscript as submitted.

Chenhao Li designed the data collection instruments, collected the data and approved the final manuscript as submitted.

Haipeng Zhang collected the data, reviewed and revised the manuscript and approved the final manuscript as submitted.
